The article "Construction of Cognitive Model of Family Education Decision-Making Based on Neural Network" was retracted in 2023. Reasons: signs of a paper mill; suspected computer-generated content; unreliable results or conclusions; concerns about the data.

# Construction of Cognitive Model of Family Education Decision-Making Based on Neural Network

**DOI:** 10.1155/2022/4082381

**Published:** 2022-07-05

**Authors:** Wenwen Yao, Ying Zhen, Yu Zhang

**Affiliations:** School of Educational Science, Mudanjiang Normal University, Mudanjiang, Heilongjiang 157011, China

## Abstract

Family's academic cognition influences the family's academic concept, rearing fashion, and academic participation. It is no longer solely associated to kid's bodily and intellectual development; however, additionally associated to household concord and social progress. With the development of the times, the complicated traits of training proceed to pose new challenges to parents. Exploring the composition and operation mechanism of family training decision-making cognition is envisioned to stop up the key to promote parents' orderly coaching participation and home university cooperation. However, the associated lookup of usual cognitive mannequin has terrible steadiness and prediction charge in focus results. This paper constructs a cognitive model of family training decision-making principally based totally on neural network. Through the assessment of relevant data, they have an effect of the cognitive model of family coaching decision-making mainly based totally on neural neighborhood evaluated from the accuracy, root suggest rectangular error RMSE, and AUC curve. The experimental effects exhibit that the prediction accuracy of the cognitive mannequin of household training decision-making primarily based on neural community is 15% greater than that of the standard model, and the cognitive balance of the mannequin is 8.2%. This paper demonstrates the effectiveness, feasibility, and practicability of the mannequin in realistic teaching.

## 1. Introduction

Education is the cornerstone of countrywide rejuvenation and social progress and the vital way to enhance countrywide nice and promote people's all-round development. The imperative motive of schooling is to instruct certified skills for the use of the society. With the development of society and the improvement of science and technology, it is challenging for the college students skilled by using common schooling to have the potential required by using state-of-the-art society. The modern-day college instructing mannequin is a long way from the thought of student-cantered. Teachers normally train dozens or even heaps of human beings in the class, which is hard to hold close the cognitive difficulties of scholar companies and persons in time and precisely and information college students to learn [1]. This frequently leads to the accumulation of students' problems, which is challenging to maintain up with the educating growth and can no longer be utterly developed. Today's society attaches outstanding significance to education. Now, people now no longer entirely pay pastime to students' take a look at rankings or ranking in the school and, alternatively, moreover, hope to reap diagnostic facts about students' cognitive structure and getting to be aware of conceivable via the test, to objectively reflect consideration and cure college students [2]. Some specialists and students have known as for the reform of the modern-day instructional examination techniques on many occasions. The ministry of training noted in the applicable coverage files that the way of academic examination and comparison must be reformed to supply full play to the cognitive diagnostic characteristic of examination.

Educational cognition is the beginning factor of subject's instructional participation. The stage of subject's academic cognition restricts the diploma of subject's academic participation and the incidence of instructional behaviour [3]. The subject's fine cognition in line with the fact and the subject's improvement fashion is the warranty of wholesome and harmonious academic participation and development [4]. Without right academic cognition, energetic and high-quality academic participation cannot be formed. In this sense, instructional cognition is absolutely the principal premise of academic participation. The alternate of academic cognition can lead to the exchange of subject's academic participation [5]. In most cases, the acquisition of this educational cognition does now no longer come from the hold close of the desirable rationality of college training and, however, the result of the routine tendency normally popular with the aid of dad and mom primarily based on the ride of social organizations and the inheritance of ordinary culture. The search on parents' academic questioning and tutorial behavior broadly speaking focuses on the awesome educational thoughts at the again of different academic participation and in the main explores its influencing elements from the social stratification concept and cultural capital theory [6]. However, the appreciation of parents' academic participation and its present troubles is nonetheless superficial, and there is no actual perception into the troubles of academic cognition as a hidden factor. The assessment outcomes of the standard cognitive decision-making mannequin in accuracy, root imply rectangular error RMSE, and AUC curve are 55% accuracy and 73.2% stability. There is nevertheless a lot room for enchantment and improvement.

This paper constructs a cognitive mannequin of household training decision-making primarily based on neural network. The experimental effects exhibit that the prediction accuracy of the cognitive mannequin of household schooling decision-making primarily based on neural community is 15% greater than that of the standard model, and the cognitive balance of the mannequin is 8.2% higher. It demonstrates the effectiveness, feasibility, and practicability of the mannequin in realistic teaching. The organizational shape of the paper is as follows: Section 1 is the introduction. This paper quickly describes the lookup background, reason, and value of the cognitive mannequin of household training decision-making based totally on neural network.  Section 2 discusses the associated work and analyses the lookup repute of choice cognition and utility at domestic and abroad.  Section 3 is associated principles and theories. Neural network, cognitive prognosis concept, and cognitive mannequin based totally on neural community are introduced.  Section 4 is the utility case and impact analysis. The accuracy of cognitive consequences and the real-time of analysis are analysed.  Section 5 is the conclusion and prospect. This paper summarizes the innovation and conclusion of this study, displays on the shortcomings of the research, and places ahead the issues that want similarly lookup in the future.

## 2. Related Work

In phrases of the theoretical foundation of cognitive development, many pupils have additionally mentioned it from distinct angles. For example, discover the concern of cognitive improvement from the element of physiological basis. This paper discusses cognitive improvement based totally on the improvement of genius shape and function. Other students additionally commenced to attempt to set up the computational mannequin of cognitive improvement from the standpoint of synthetic neural network. Some humans labelled it into neural constructivism or cognitive neuropsychology. Relevant research is summarized as follows:

Piaget's principal researches the established hassle of kid's cognitive development. Applying it to adolescents with incredible talent and reading the regulation of kid's cognitive increase in the new educating surroundings suggest some limitations. As for how to prolong it to the problem of person cognitive development, some authors are additionally involved [7]. After adults, there are many elements worried in the trouble of cognitive development, and the in-depth learning about of this situation by way of some different theories is additionally instructive, for example, the idea of fluid brain and crystal genius proposed by means of cartel and others [8]. Other authors have additionally tried to discover the neurophysiological mechanism of universal fluid talent 48%. It indicates that we can habit in-depth look up on cognitive improvement at a greater primary level. The complexity of cognitive boom lookup is additionally mirrored in the challenge of experimental operation. Although there are many superior applied sciences that can assist researchers find out about human psychology, it is nonetheless tough to attain a very correct quantitative evaluation like physics [9]. Due to the particularity and complexity of education, household schooling decision-making cognition, as an educational and expert psychological field, has now not been paid interest to by means of pupils at domestic and overseas for a lengthy time. The present applicable literatures lookup consequences on the whole focal point on the utility of household training theory, gadget theory, price theory, feature theory, schooling methodology, and different theories. Most of them deduce parents' academic cognition based totally on parents' academic behaviour or analyse the guiding position of cognitive elements on instructional behaviour [10]. Overall, these recommended explorations lack the simple theoretical and theoretical integrity in the discipline of cognitive problems, omit the incomparable balance traits of instructional cognition itself, and bypass the linkage traits of academic cognition as a psychological process. The most vital aspect is that there is a deviation in the underlying common sense when dad and mom analyse instructional problems. They frequently research from overseas instructional trip or instructional idea publicized by means of the media and primarily based on their personal trip to understand, internalize, practice, and expand, and even create new knowledge, which will inevitably lead to misunderstanding, misuse, or indigestion. The cognition of the essence of education, that is, what is education, what is the use of education, and how schooling must be done, is indistinct and fragmented.

More and greater interest has been paid to the trouble of exploring cognitive improvement thru synthetic neural community theory. This vital lookup course of neural community is referred to as cascade correlation model. The neurons of this neural community will develop overtime and reap a quicker studying velocity than the error again propagation algorithm [11]. At present, some authors use neural community mannequin to discover the troubles of cognitive improvement and person differences, whilst others establish neural community mannequin to simulate the phased traits of cognitive development. In addition, many fashions have been set up to behaviour in-depth look up on a number subsubjects associated to cognitive growth [12]. These fashions encompass the neural community mannequin of grownup talent injury, the regular mannequin of child cognitive development, the labelled gaining knowledge of mannequin of early infants, the computational evaluation mannequin of conservation, the neural community mannequin of kid's perceptual development, the neural community mannequin of kiddies obtaining the ideas of distance, time, and speed, the neural community mannequin of early reminiscence development, the neural community mannequin of cognitive improvement disorder, etc. This sort of literature primarily focuses on how to use computational fashions to simulate Piaget's idea of 4 levels of kid's cognitive development.

## 3. Related Theories and Technologies

### 3.1. Neural Network Model

Neural community is a computing shape that displays the traits of human brain. It is a manner of simulating human genius on the groundwork of current neurobiology research. It is solely the abstraction, simplification, and simulation of human intelligence anxious machine to a positive extent, as a substitute than the actual description of human talent apprehensive system [13]. According to the fundamental shape and characteristic of organic neural network, neural community is composed of neurons and their nerve endings. Therefore, to simulate organic neural network, we first want to simulate organic neurons. Neural networks typically name neurons processing units, and every so often, they can be known as nodes from the viewpoint of networks. Artificial neuron is the simple facts processing unit of neural community operation. It abstractly describes the statistics processing technique of organic neurons with mathematical language and describes its simulation shape and characteristic with mannequin diagrams.

With the speedy improvement of synthetic brain technology, neural community has attracted extremely good attention, frequently due to the fact that neural community has the following advantages: first, mechanically acquire the legal guidelines contained in samples and can gain nonlinear output with arbitrary accuracy. Second, the data is evenly disbursed and saved in every neuron in the network, so the neural community has appropriate fault tolerance and robustness [14]. Thirdly, it has self-adaptive ability; through self-learning of the exterior environment, the neural community can reconstruct its interior organization. Fourth, associative reminiscence for exterior stimuli or inputs. Fifth, the use of the dispensed processing method: we can shortly discover the superior solution. The sturdy potential of neural community to resolve complicated troubles makes it greater and extravalued by means of researchers.

The neural community is composed of output layer and output layer. The enter layer includes *n* neurons for inputting data. The neurons in the output layer are organized in a range of ways, which include one-dimensional linear array and two-dimensional airplane linear array, as proven in Figure 1. The neurons of the output layer and the neurons of the enter layer are linked with the aid of the weight vector, and each neuron of the output layer obtains the likelihood to reply to the enter data of the enter layer through competition. It can mechanically locate the inner legal guidelines and integral attributes in the samples and self-organizing and adaptive exchange of the community parameters and structure [15]. It can elevate out unsupervised aggressive learning, which is comparable to the mastering manner of organic neural community in human brain. The neural community can adaptively modify the community weight in accordance to the samples, so that every neuron in the output layer is solely touchy to the unique enter sample class, and its internal megastar weight vector turns into the core vector of the sample class, that is, the clustering centre. This self-organizing clustering technique can mechanically classify the enter samples besides specifying the anticipated output.

### 3.2. Construction of Cognitive Development Model

Based on the above theoretical basis, this paper constructs a mannequin of cognitive development. The mannequin is often based totally on neural community theory and, however, additionally considers the expertise of some different disciplines. For a neural community system, there are quite a few necessary parameter variables: the range of neurons, the wide variety of connections between neurons, computational complexity, cognitive mode, cognitive depth, and different parameters interact, which immediately influence the procedure of cognitive development.

(1) $$\begin{array}{c} \frac{dI\left(t\right)}{dt}=\frac{\alpha I\left(t\right)}{I{\left(t\right)}^{2}}-\left[\frac{I\left(t\right)}{A}+\beta \right]. \end{array}$$

The solution of logistic equation is:

(2) $$\begin{array}{c} I\left(t\right)=\frac{\left[\left(I\left(t\right)/A\right)+\beta \right]}{{me}^{-at}}+\frac{\alpha I\left(t\right)}{I{\left(t\right)}^{2}}. \end{array}$$

The cognitive sample corresponds to the reminiscence sample or reminiscence potential of a neural network. For utterly interconnected Hopfield neural networks, there is a higher restrict on the cognitive mode of neural networks. Generally, the following relationship is satisfied:

(3) $$\begin{array}{c} M\left(t\right)\leq 0.15I\left(t\right). \end{array}$$

In addition to the influence of the number of neurons on cognitive patterns, the decline of the function of the whole neural network system will also affect the change of the number of cognitive patterns. The decline of neural network function leads to the decrease of memory capacity of neural network. The decline of neural network function may be manifested in two aspects. On one hand, it leads to the discount of the quantity of neurons and the range of connections between neurons. On the other hand, it leads to the weakening of the characteristic of neurons and the connections between neurons. The connection function between neurons is weakened, resulting in the weakening of the signal of nerve impulse. In order to simplify consideration, the effect of this recession on memory capacity can be described in the form of index:

(4) $$\begin{array}{c} M\left(t\right)=\frac{0.15I\left(t\right)}{e^{-g\left(t\right)}}+{me}^{-\alpha t}+c. \end{array}$$

In realistic application, the overall performance of neural community is now not perfect, and it regularly fails in training. With the growing complexity of the mannequin and extending wide variety of hidden layers, the records primarily based on time collection with massive span of neural community is tough to be processed rapidly and accurately. This is due to the fact that the product of Jacobian matrix modifications is great. As a result, neural community is challenging to deal with records with massive span [16]. In gradient learning, there is a quantitative relationship between the mannequin parameter zero and the loss feature *L*. In essence, the distinction between the expected price and the real cost is used as the loss feature value, in order to reduce the loss characteristic value. Finally, the gradient facts are calculated in accordance to the loss function, which is again to the coaching mannequin parameters and modified accordingly. Through some transformation, it corresponds to the nation of the subsequent second one with the aid of one. The mathematical expression of the gradient of the loss feature *L* with appreciate to the parameters at time *t* is proven in

(5) $$\begin{array}{c} \frac{\partial L_{T}}{\partial \theta }=\frac{\sum_{t\leq T}\partial L_{T}/\partial S_{T}\cdot \partial F_{T}\left(x,y\right)/\partial \theta }{\left(S_{t-1},x_{t}\right)-\left(x,y\right)}. \end{array}$$

According to the chain rule, decompose the matrix as shown in

(6) $$\begin{array}{c} \frac{\partial S_{T}}{\partial S_{T}}=\frac{\left(\partial F_{T}\left(x,y\right)/\partial \theta \right)\left(\partial F_{T}\left(x_{t-1},y\right)/\partial \theta \right)\left(\partial F_{T}\left(x_{t-2},y\right)/\partial \theta \right)\cdots \left(\partial F_{T}\left(x_{1},y\right)/\partial \theta \right)}{\varphi_{1}+\varphi_{2}+\cdots +\varphi_{t}}. \end{array}$$

Cognitive diagnostic evaluation is to supply inexperienced persons or instructors with diagnostic statistics about learners' mastering kingdom on the foundation of trying out learners, that is, learners' mastery of understanding points. The cognitive analysis mannequin believes that there is an interior relationship between learners' mastery of expertise factors and learners' rankings on workout routines and the relationship between matters and understanding points [17]. By the usage of learners' studying report coaching model, learners' ratings on new subjects can be predicted. Figure four indicates the precise waft of the cognitive analysis model. Process analysis of cognitive diagnosis is shown in Figure 2.

### 3.3. Construction of Cognitive Model of Family Education Decision-Making

Educational cognition lookup is no longer solely a cognitive result and, however, additionally desires to wholly think about the procedure and linkage of academic cognition as a one-of-a-kind social cognition. This manner and linkage mark the cognitive stage of household schooling decision-making [18]. The 4 dimensions of academic knowledge, instructional value, academic ride, and instructional decision-making are of extraordinary magnitude to analyse the cognitive degree of education. These 4 dimensions exhibit a modern and cyclic relationship between stimulation and behavioural response patterns. Each cycle will deepen the cognitive subject's cognition and grasp of college instructional expertise and instructional value and, in the end, internalize the perceived and skilled college schooling in the psychological shape of the cognitive subject, forming a new instructional judgment and decision-making, which constitutes a hierarchical shape for measuring the degree of instructional cognition; educational expertise and instructional price are nearer to stimulation, whilst instructional ride and instructional decision-making are nearer to behavioural response.

All the cognitive effects of parents' faculty education, whether empirical or conceptual, must be viewed as academic knowledge. In this sense, academic know-how is the simple way and rules of household training decision-making cognition. Educational know-how lays the basis of instructional cognition. The attribution essence of training is the simple aspect of instructional knowledge. It is the essence of academic information specific from different popular human cognition, which by and large entails the descriptive proposition of what it is. The manner attribute of schooling is the content material of sensible things to do that permeate the instructional world and the social world. It implies the procedural operation in the technique of instructional cognitive construction, in the main involving the procedural proposition of how to do. Understanding the nature of schooling is the premise of organising the attribute of academic process [19]. The approach attribute of cognitive coaching is moreover the usage of stress to apprehend the essence of education. The nature and system attribute of appreciation and cognitive training can promote the difficulty to reconstruct the genuine which means of schooling on the groundwork of the unique social experience, which is, by way of no skill an easy extension of repeated academic meaning, however, a procedure of unconscious and unconscious academic cognition and understanding. Educational cognitive model was shown in Figure 3.

Educational fee is really parents' subjective creativeness and expectation of college education, which impacts our academic cognition to a top-notch extent. It is a customary cognitive nation when we deal with academic records and instructional events. Combined with the present lookup on academic cognition, on the foundation of defining the cognition of household training decision-making, this paper determines the 4 dimensions of academic knowledge, instructional value, academic journey, and instructional decision-making, involving what faculty schooling is, what use college training is, the relationship between faculty training and household education, and how we need to intervene in instructional activities [20–22]. The above 4 dimensions have developed into successively circulating instructional cognitive hyperlinks in instructional activities. Make mannequin assumptions from the following three stages; educational cognition is an exclusive social cognitive exercise carried out with the aid of dad and mom for the individualized and socialized improvement of their children. It is a cost cognition primarily based on the wants of sure subjects. Educational charge is developed via mom and father for the sake of the relationship between kid's future development, taking wishes and their very very own pastimes as the commencing point, taking the significance and rate of the beneficial attributes of education to parents, and discovering and in search of educational value in the approach and on the basis of producing educational knowledge. After all, the instructional information we shape in the instructional world is influenced with the aid of our dreams and values.

## 4. Experiment and Analysis

From the elements of classification and regression, the contrast indicators, together with accuracy, root imply rectangular error RMSE, and AUC curve, are used to consider the impact of the cognitive mannequin of household training decision-making based totally on neural network.

### 4.1. Analysis of Knowledge Cognition Effect

Figure 4 suggests the prediction effects of the cognitive analysis mannequin that solely will increase the significance of understanding factors and the velocity of doing questions on learners' scores. Math 1 and math 2 have a small quantity of data and help incorporates a giant quantity of data. However, it can be virtually considered from the desk that on the three facts sets, the prediction accuracy of the cognitive mannequin of household schooling decision-making primarily based on neural community is greater than that of the different 5 cognitive analysis models, and it additionally has higher stability. It suggests that the software of two factors, the significance of expertise factors and the velocity of doing questions, to the cognitive prognosis mannequin can enhance the analysis effect.

Figure 5 is the change curve of loss function value and RMSE value between the cognitive model of family education decision based on neural network and the traditional cognitive model on three data sets.

As can be viewed from Figures 5(a) and 5(b), on math 1 and math 2 records sets, the loss characteristic cost of the cognitive mannequin of household training decision-making based totally on neural community is greater than that of the standard cognitive model; however, on the aid statistics set, the loss feature fee of the cognitive mannequin of household training decision-making primarily based on neural community is greater stable, indicating that including parameters affecting studying can make the mannequin higher simulate the mastering process. It can be viewed from Figures 5(c) and 5(d) that the two fashions first decline and then upward push on the three statistics sets, and the minimal price is about 1 epoch. However, in distinction with the normal cognitive model, the RMSE of the neural network-based family coaching decision-making cognitive model on math 1 and math 2 data gadgets is usually lower, indicating that the neural network-based family coaching decision-making cognitive model has greater stability. The help fact set is no longer as low as the ordinary cognitive model, due to the fact that the quantity of help records is larger, which makes the mannequin coaching greater mature.

Figure 6 is the change curve of prediction accuracy and ROC between the cognitive model of family education decision based on neural network and the traditional cognitive model on three data sets.

As can be viewed from Figures 6(a) and 6(b), the two fashions upward thrust and then fall on the three information sets, indicating that the mannequin can acquire optimization after education 2-4 epochs. On the three records sets, the prediction accuracy of the cognitive mannequin of household schooling decision-making primarily based on neural community is barely decreased than that of the regular cognitive model; however, the prediction accuracy of the cognitive model of household training decision-making primarily based on neural community is extramalleable. The ROC curve of the household training choice cognitive mannequin primarily based on neural community is nearer to the higher left nook on math 1 information set, whilst it is equal on the different two statistics sets, indicating that the amplification of the significance of understanding factors and the velocity of doing questions have a positive influence on the model.

### 4.2. Comparison of Pretest Differences between Experimental Group and Control Group

Figure 7 suggests the prediction effects of the cognitive prognosis mannequin after education on learners' scores. It can be considered from the desk that on the three record sets, the prediction accuracy of the cognitive mannequin of household training decision-making primarily based on neural community is greater than that of the different 5 cognitive prognosis models; however, it is comparable to that of the ordinary model. It suggests that the utility of neural community mannequin to cognitive prognosis mannequin can improve the prognosis effect; however, it is distinctive from that affecting the gaining knowledge of effect.

Figure 8 is the change curve of the loss function value and RMSE value of the family education decision cognitive model based on neural network and the other two neural networks on three data sets.

As can be considered from Figure 8, the loss characteristic fee of the cognitive mannequin of household schooling selection based totally on neural community is lower than that of the different two models, indicating that the getting to know capacity of the cognitive mannequin of household training selection primarily based on neural community is stronger. The minimal price and suggested cost of the cognitive mannequin of household training selection primarily based on neural community on the three records units are much less than the different two models, indicating that the cognitive mannequin of household schooling choice primarily based on neural community has higher stability. On the statistics units math 2 and assist, the accuracy of the cognitive mannequin of household schooling decision-making based totally on neural community is distinctly high; however, on math 1, it is greater than the regular mannequin in the early stage and decreases than the typical mannequin in the later stage, which in addition indicates that the cognitive mannequin of household training decision-making based totally on neural community has more advantageous studying ability. The ROC curve of the cognitive prognosis model that totally changes the neural neighborhood is extended in three statistics gadgets in distinction with the frequent cognitive model; alternatively, it is no longer as proper as the everyday effect, indicating that the effect of getting to understand factors on the prognosis model is greater than that of the neural neighborhood model.

## 5. Conclusion

In this paper, a cognitive mannequin of household training decision-making primarily based on neural community is proposed. It combines neural community to analyse complicated motor interactions in order to acquire correct and interpretable diagnostic results. In the technique of education and inspecting the information set, this finding acquired the learners' mastery diploma and expertise stage of distinct understanding points and performed exact effects in prediction accuracy. This will assist educators higher recognize learners' expertise stage and formulate dynamic educating strategies, to enhance educating efficiency. The cognitive model of family training decision-making primarily based completely on neural neighborhood simulates the elaborate interaction machine between freshmen and practice, avoids the problems of many neural neighborhood parameters and gradient disappearance, and is higher in line with the qualities of learners' time sequence primarily based completely learning. This paper places ahead the cognitive mannequin of household schooling decision-making based totally on neural network. Although it breaks via the discrete features of traditional cognitive model and will enlarge the influencing factors affecting learners' gaining understanding of effect, the selection of neural neighborhood model desires to be in addition improved. Because the getting to know procedure is affected by means of many aspects, the influencing elements are nonetheless perfect. Through the lookup on the cognitive mannequin of household training decision-making primarily based on neural network, the verifiability contrast is carried out, and the lookup effects are anticipated to have in addition guiding value for instructional practice.

## Figures and Tables

**Figure 1:** Output matrix of neural network.

**Figure 2:** Process analysis of cognitive diagnosis.

**Figure 3:** Educational cognitive model.

**Figure 4:** Prediction results of learners' performance in different models.

**Figure 5:** Loss value and RMSE value of different cognitive models on three data sets.

**Figure 6:** Prediction accuracy of different models on data sets.

**Figure 7:** Loss value and RMSE value of different cognitive models on three data sets.

**Figure 8:** Curves of different cognitive models on math data set.

## Data Availability

All data, models, and code generated or used during the study appear in the submitted paper.
